The article "CDK5 Mediates Proinflammatory Effects of Microglia through Activated DRP1 Phosphorylation in Rat Model of Intracerebral Hemorrhage" was published in 2022. Journal: Dis Markers.

# CDK5 Mediates Proinflammatory Effects of Microglia through Activated DRP1 Phosphorylation in Rat Model of Intracerebral Hemorrhage

**DOI:** 10.1155/2022/1919064

**Published:** 2022-06-27

**Authors:** Mingqing He, Xiaoyan Wang, Zheng Liu, Qiyuan Cui, Ying Chen, Wenqing Geng, Jinzhou Zhu, Jiabing Shen

**Affiliations:** ^1^Department of Geriatrics, The First Affiliated Hospital of Soochow University, Suzhou, Jiangsu Province, China; ^2^Key Laboratory for Aging & Disease, Nanjing Medical University, Nanjing, Jiangsu Province, China; ^3^Department of Respiratory Medicine, Affiliated Hospital of Nantong University, Nantong, Jiangsu Province, China; ^4^Department of Endocrinology and Metabolism, The First Affiliated Hospital of Soochow University, Suzhou, Jiangsu Province, China; ^5^Department of Neurology, Affiliated Hospital of Nantong University, Nantong, Jiangsu Province, China; ^6^Department of Gastroenterology, The First Affiliated Hospital of Soochow University, Suzhou, Jiangsu Province, China

## Abstract

**Introduction:**

Cyclin-dependent kinase-5 (CDK5) is a key kinase involved in brain development and function and recently found to be involved in neuronal and astroglial apoptosis, neural stem/progenitor cell stemness, mitochondrial fission, and synaptic transmission. But the specific mechanism of CDK5-mediated anti-inflammatory remains unclear in ICH. The aim of the present study was to explore the role of CDK5 in mediating microglia activity through activated DRP1 phosphorylation in a rat ICH model.

**Methods:**

We measured behavioral change after ICH; detected the expression of CDK5 in the rat brain using immunohistochemistry; and measured the protein levels of CDK5, p35, p25, p-histone H1, and p-DRP1 using Western blot analysis. Coimmunoprecipitation analysis indicated interaction of CDK5 and DRP1. Tumor necrosis factor-*α*, interleukin- (IL-) 1*β*, and IL-6 levels were measured using enzyme-linked immunosorbent assay (ELISA).

**Results:**

After ICH, CDK5 protein level and kinase activity increased. Western blot data showed that CDK5 expression increased from 6 h and peaked at 2 d after ICH (*p* < 0.05), and the expression of p35 was lowest at 12 h, while the expression of p25 peaked at 2 d after ICH. Besides, p-DRP1 expression change follows with CDK5 kinase activity change. Coimmunoprecipitation showed that interaction between CDK5 and DRP1 certainly exists in microglia. Then, knockdown CDK5 or p35 expression by siRNA reduced the expression level of p-DRP1. ELISA data showed that the protein levels of proinflammatory mediators, such as TNF-*α*, IL-1*β*, and IL-6, were decreased by knockdown of CDK5.

**Conclusion:**

CDK5 may regulate DRP1 by direct phosphorylation in microglia and further induce microglia secreting proinflammation factor.

The article "CDK5 Mediates Proinflammatory Effects of Microglia through Activated DRP1 Phosphorylation in Rat Model of Intracerebral Hemorrhage" was published in 2022. Journal: Dis Markers.

## 1. Introduction

Intracerebral hemorrhage (ICH) is a subtype of stroke with high mortality and morbidity. The prevalence of ICH in the elderly is increasing rapidly, and this disease seriously endangers the health and life of elderly patients [1]. When the arteries in the brain rupture, the hematoma triggers a series of physiological and pathological reactions, which can cause primary and following brain damage [2].

Microglia are extremely important for hematoma and debris clearance, but hyperactivation is also a factor in secondary inflammation in ICH [3]. Microglia are resident macrophages of the central nervous system. They have the function of phagocytizing cell debris, presenting foreign antigens, and are sensors of pathological events including ICH [4]. After ICH happens, microglia are activated in a short period of time. Activated microglia play a phagocytic effect by removing hematoma and damaged cell debris, thereby protecting nerve cells and providing a favorable environment for the recovery of ICH [5, 6]. However, the excessive activation of microglia can release various cytokines, chemokines, nitric oxide, free radicals, and other potentially toxic chemicals, triggering and aggravating the brain damage induced by ICH [5]. The release of proinflammatory mediators can induce the infiltration of inflammatory cells, such as leukocytes and macrophages, thereby exacerbating neurological deficits [7, 8].

CDK5 is a unique member of cyclin-dependent kinase (CDK) family and is activated by p35 and p39 [9]. Unlike other members of the CDK family, CDK5 is not involved in cell-cycle progression [10]. During calcium homeostasis dysregulation, calcium-dependent calpains can proteolytically hydrolyze p35 and p39, resulting in the formation of p25 and p29. Mutant proteins p25 and p29 are stripped of their membrane anchoring sequences, which will lead to relocation of the active CDK5 complex, resulting in aberrant activation of CDK5, which has been confirmed in many neurotoxic diseases, such as Alzheimer's disease, Parkinson's disease, cerebral ischemia, and neurodegenerative diseases [11–13]. As a protein kinase, its function is always associated with phosphorylating various kinds of downstream substrates in cells [13]. CDK5, which binds to p25, is thought to be deregulated to produce highly phosphorylated tau protein and destroy the cytoskeleton of neurons [12]. In our previous study, CDK5 upregulate in ICH and promote neuronal apoptosis by phosphorylating transcription factor MEF2D [14]. In addition, DRP1 is a protein associated with mitochondrial fission, which can be phosphorylated by CDK5 in neuron; the exact role is not clear in ICH [15].

The article "CDK5 Mediates Proinflammatory Effects of Microglia through Activated DRP1 Phosphorylation in Rat Model of Intracerebral Hemorrhage" was published in 2022. Journal: Dis Markers.

In recent studies, CDK5 demonstrated an ability to fine-tune inflammation responses. For example, in BV2 cells, activated cyclin-dependent kinase 5 promotes the phagocytosis of fibrillary *β*-amyloid by microglia by upregulating the expression of lipoprotein lipase [16]. What is more, mitochondrial fission can urge the microglia secrete proinflammatory factor [17]. In a conclusion, we found that CDK5 can regulate DRP1 by phosphorylation in microglia and further induce microglia secreting proinflammation factor.

## 2. Materials and Methods

### 2.1. Experimental Animals and ICH Model

Experiments were performed based on the National Institutes of Health Guidelines for the Care and Use of Laboratory Animals published by National Research Council in 1996. Male Sprague-Dawley rats (230-260 g) in this study were approved by the Department of Animal Center and Use Committee in Nantong University (ethical approval number: 20160906001). Animals were housed five per cage under a 12 h light/12 h dark cycle and at constant temperature (24°C) with sufficient food and water. ICH model was used as the previously described with minor changes [9]. The animals were divided into two groups, sham and ICH groups. First, rats were anesthetized by intraperitoneal injection of a mixture containing ketamine (100 mg/kg; Sigma-Aldrich, St. Louis, MO) and xylazine (10 mg/kg; 2 : 1 *v*/*v*; Sigma-Aldrich). Then, autologous whole blood was collected by putting the tail tip in warm water for 3-4 min, cleaning the skin with 75% alcohol, cutting the tail tip, and drawing 50 *μ*l of freely dripping blood into a sterile syringe. Autologous whole blood (50 *μ*l) was infused into the right caudate nucleus stereotactically (coordinates: 0.2 mm anterior, 5.5 mm ventral, and 3.5 mm lateral to the bregma) using a microinjector at a rate of 5 *μ*l/min through a 26-gauge needle. The needle was removed 10 min after injection, and then, closed the skin incision. The sham group performed the same operation but only received a pause of microinjector for 20 minutes without autologous blood injection. After the surgery, the rats were housed in a 24°C room and had free access to food and water after waking up from anesthesia. For Western blot analysis of brain extract, the ICH group and the sham group were sacrificed to extract the brain protein at 3 h, 6 h, 12 h, 1, 2, 3, 5, and 7 days following ICH.

### 2.2. Forelimb Placing Test

The rats were held by their torsos in order that the forelimb could hang free, which referred to our previous studies [14]. Independent testing of each forelimb was given rise to brushing the respective vibrissae on the corner edge of a countertop. Intact animals put the forelimb quickly onto the countertop. In the light of the extent of injury, placing of the forelimb contralateral to the injury may be impaired. In the process of experiments, each rat was tested ten times for each forelimb, and the percentage of trials in which the rat placed the left forelimb was counted.

The article "CDK5 Mediates Proinflammatory Effects of Microglia through Activated DRP1 Phosphorylation in Rat Model of Intracerebral Hemorrhage" was published in 2022. Journal: Dis Markers.

### 2.3. Corner Turn Test

The corner turn test was conducted with minor revise to our previous studies [14]. The rats were allowed to enter into a corner, the angle of which was 30°C. To exit the corner, the rat should turn either to the left or to the right. Only the turns involving full rearing along either wall were included. According to the extent of injury, rats may show a tendency to turn to the side of the injury. The percentage of right turns was scored as the corner turn score. The trial was repeated 10 times and at least 30 s interval for each trial.

### 2.4. Western Blot Analysis

To obtain samples for Western blotting, rats were sacrificed at different time points (*n* = 5 for each time point) by giving overdose of containing ketamine and xylazine, and the brain tissues surrounding the hematoma (extending 4 mm to the hematoma) as well as an equal part of the normal, sham-controlled, and contralateral tissue were excised and snap frozen at −80°C until use. In order to prepare lysates, frozen caudate put amen tissue samples were weighed and minced with eye scissors in ice and then homogenized in lyses buffer (50 mM Tris, pH 7.5, 5 mM EDTA, 1% SDS, 1% sodium deoxycholate, 0.1% Triton X-100, 1 mM PMSF, 10 *μ*g/ml aprotinin, and 1 *μ*g/ml leupeptin) and clarified by centrifuging at 12,000*g* for 20 min in a microcentrifuge at 4°C. After determination of its concentration with the Bradford assay (Bio-Rad), the resulting supernatant was subjected to SDS-polyacrylamide gel electrophoresis (PAGE); proteins were transferred to a polyvinylidene difluoride (PVDF) membrane (Millipore) by a transfer apparatus. Then, the membrane was blocked with 5% nonfat milk for 2 h and incubated with primary antibody against CDK5 (anti-mouse, 1 : 1000; Santa Cruz), DRP1 (anti-rabbit, 1 : 1000; Santa Cruz), p-DRP1 (anti-mouse, 1 : 500; Cell Signaling), and GAPDH (anti-rabbit, 1 : 1000; Sigma) at 4°C overnight. At last, the membranes were incubated with a second antibody, and protein was visualized using an enhanced chemiluminescence system (Pierce Company, USA).

### 2.5. Sections and Immunohistochemistry

Rats from 2 days after ICH or sham group were anesthetized and perfused with 500 ml of 0.9% saline, followed by 4% paraformaldehyde in 0.1 M phosphate-buffered saline (PBS), pH 7.4 (supplied by Solarbio® Life Sciences). After that, the brains were removed, post fixed in the same fixative overnight at room temperature (RT), and subsequently replaced with 20 and 30% sucrose for 2-3 days, respectively. The tissues were then cut at 5 *μ*m with a cryostat, and the sections were stored at −20°C until use. For immunohistochemistry, brain sections were washed briefly in phosphate-buffered saline (PBS) and then treated with 3% H_2_O_2_ for 10 min at RT to reduce endogenous peroxidase activity. After that, the sections were incubated with blocking solution and reacted with an anti-CDK5 antibody and subsequent secondary antibody. The sections were color-reacted with the liquid mixture (0.02% diaminobenzidine tetrahydrochloride (DAB) and 3% H_2_O_2_). Finally, the sections were air-dried, dehydrated, covered with coverslips, and examined using a Leica microscope (Germany).

The article "CDK5 Mediates Proinflammatory Effects of Microglia through Activated DRP1 Phosphorylation in Rat Model of Intracerebral Hemorrhage" was published in 2022. Journal: Dis Markers.

### 2.6. Immunoprecipitation

BV2 microglia (cultured with DMEN with 10% fetal bovine serum (FBS) supplement, which purchased from National Collection of Authenticated Cell Cultures, Shanghai, China) were promptly homogenized in lysis buffer and then centrifuged at 12,000*g* at 4°C for 20 min to collect the supernatant. Immunoprecipitation was performed by incubating 0.5 mg of total cell lysates with anti-CDK5 (anti-mouse; Santa Cruz) or anti-DRP1 (anti-rabbit; Santa Cruz) primary antibody at 4°C overnight. Protein G-Sepharose (Sigma, 1 : 1 slush in PBS) was then added at 4°C wheel rocking for 2 h. The precipitates were washed four times with ice-cold PBS, resuspended in 50 *μ*l 2× SDS sample buffer, and boiled for 5 min at 100°C. Finally, Western blot analysis was conducted as described above.

### 2.7. RNA Interference

BV2 cells grown in 12-well plates for 24 h were transfected with siRNAs against target genes (5′-ACGTGGTCTTCCTCTACAT-3′, p35/25 siRNA: sc-35047; Santa Cruz Biotechnology, USA) or control siRNA (5′-ACGUGACACGUUCGGAGAATT-3′, sc-37007, Santa Cruz Biotechnology, USA) with lipofectamine 2000 (Invitrogen). At 24 h posttransfection, cells were treated with 30 *μ*M hemin at 37°C for 0.5 h, and then, culture supernatants and cells were harvested for the subsequent experiments.

### 2.8. Assays for CDK5 Activity

Phosphorylation of histone H1 by activated CDK5-associated kinase activity was carried out as previously described with some modifications [14]. Briefly, CDK5 was immunoprecipitated from the brain homogenates using an anti-CDK5 antibody conjugated to agarose beads (C8; Santa Cruz Biotechnology). Immune complexes precipitated with anti-CDK5 antibody were washed two times with PBS and resuspended in 50 *μ*l kinase buffer (50 mM Tris-HCl, pH 7.2, 10 mM MgCl_2_, 1 mM DTT) containing 100 *μ*M ATP. One microgram of commercially purified histone H1 was then added to the immunoprecipitates, and the mixtures were incubated for 30 min at 30°C. The samples were separated by SDS-PAGE (15% polyacrylamide gels), and phosphorylated histone H1 was detected by immunoblotting with anti-phospho-histone H1-specific antibody.

The article "CDK5 Mediates Proinflammatory Effects of Microglia through Activated DRP1 Phosphorylation in Rat Model of Intracerebral Hemorrhage" was published in 2022. Journal: Dis Markers.

BV2 cells were treated with 30 *μ*M hemin for 24 h; lysed in buffer containing 50 mM Tris-HCl (pH 7.4), 150 mM NaCl, 5 mM EDTA, 1% PI, 1 mM Na3VO4, and 1 mM NaF on ice; placed on a roller at 4°C for 30 min; and then centrifuged at 14,000*g* for 15 min. The protein extracts were immunoprecipitated with an anti-CDK5 primary antibody (mouse; Santa Cruz) at 4°C for 2 h. Protein A agarose beads were added, followed by incubation for 2 h at 4°C. The beads were washed with lysis buffer and then kinase buffer (50 mM Tris-HCl (pH 7.4), 10 mM MgCl_2_, 1 mM DTT, 1 mM EGTA, and 1 mM NaF). A kinase reaction buffer consisting of 150 *μ*M ATP, 10 *μ*Ci [*γ*-32P]-ATP (specific activity: 6,000 Ci/mmol; NEN, Boston, MA), and 125 *μ*g/ml histone H1 was added to the protein samples, followed by incubation at 30°C for 30 min. The kinase reaction was then terminated by addition of 4× SDS loading buffer. Samples were boiled for 5 min and separated by 15% SDS-PAGE, and phosphorylated histone H1 was detected by immunoblotting with anti-phospho-histone H1-specific antibody (anti-mouse, 1 : 500; Cell Signaling).

### 2.9. Cytokine ELISAs

Cultured BV2 microglia were treated with hemin (30 *μ*M). Twenty-four hours after stimulation, culture supernatants were collected and centrifuged. Concentrations of TNF-*α*, IL-1*β*, and IL-6 were measured with commercially available ELISA kits (BioLegend, UK), followed by measurements in a plate reader at a wavelength of 450 nm.

### 2.10. Statistical Analysis

All data in this paper were analyzed with the Stata 8.0 statistical software. All values are expressed as mean ± SEM. The statistical analysis was determined by one-way ANOVA followed by the Tukey's post hoc multiple comparison tests. *p* < 0.05 was considered statistically significant. Each experiment consisted of at least three replicates per condition.

## 3. Result

### 3.1. The Changes of Neurological Deficits following ICH

Behavioral tests include forelimb placing test and corner turn test, which are used to measure neurological deficits in the sham operation group and the ICH group, respectively. As shown in Figure 1, compared with the sham operation group, the ICH group showed more severe neurological deficits, and there were significant differences between the two groups within the first three days.

The article "CDK5 Mediates Proinflammatory Effects of Microglia through Activated DRP1 Phosphorylation in Rat Model of Intracerebral Hemorrhage" was published in 2022. Journal: Dis Markers.

### 3.2. Immunohistochemistry Staining Exhibiting Distribution of CDK5 in the Perihematoma after ICH

Immunohistochemistry was used to identify the expression and distribution of CDK5 after ICH. Compared with the sham operation group, the number of CDK5 positive cells near the hematoma in the ICH group increased (Figure 2). The above data indicate that ICH can cause temporal changes in CDK5 protein levels, indicating that CDK5 may play a role in the process of ICH.

### 3.3. Changing Expression Level of CDK5 following ICH by Western Blot Analysis

Western blot was performed to detect the time change of CDK5 expression near the hematoma. It was found that the expression of CDK5 in the sham operation group was low, and it began to increase at 6 h after ICH and reached a peak at day 2 after ICH (*p* < 0.05) (Figures 3(a) and 3(b)). We also found the changing expression of p35/25 (Figures 3(c) and 3(d)). Our results indicated that the expression of p35 was lowest at 12 h, while the expression of p25 peaked at 2 d after ICH (*p* < 0.05).

### 3.4. The Change of CDK5 Kinase Activity and P-DRP1 Expression following ICH by Western Blot Analysis

To explore if CDK5 kinase activity changes in the rat ICH model, phosphorylation of histone H1 by activated CDK5-associated kinase activity was carried out. We found that p-histone H1 level upregulated at day 1 and reaching peak at day 3, then decreased following ICH (Figures 4(a) and 4(b)). DRP1 is a protein associated with mitochondrial fission. Previous study detected that DRP1 can be phosphorylated by CDK5 in neuron, and this can induce the increase of mitochondrial fission. Interestingly, in the rat ICH model, p-DRP1 expression change follows with CDK5 kinase activity change (Figures 4(c) and 4(d)). From the above results, we concluded that there may be a correlation between CDK5 and DRP1, but the specific mechanism is unclear.

### 3.5. DRP1 Is Phosphorylated by CDK5 in BV2 Microglia

Since most of CDK5 functions are concerned with its phosphorylation ability, and CDK5 interacts with phosphorylate DRP1 has been reported in neuron. Next, we use coimmunoprecipitation to define if CDK5 interacts with phosphorite DRP1 in microglia. The result of coimmunoprecipitation shows that interaction between CDK5 and DRP1 certainly exists in microglia (Figure 4(e)). To define if phosphorylation of DRP1 is depended on CDK5, we knock down CDK5 or p35 expression by siRNA, and data shows decrease of CDK5 or p35 reduces the expression level of p-DRP1 (Figures 4(f) and 4(g)).

### 3.6. DRP1 Phosphorylated by CDK5 Promote the Expression Proinflammatory Mediators

In the past research, mitochondrial fusion and fission are mentioned in maintaining mitochondrial functions including mitochondrial biogenesis and distribution as well as apoptosis, cell division, and complementation of mitochondrial DNA [15]. Park et al.'s research indicates that the phosphorylation of DRP1 is responsible for the increased expression of proinflammatory mediators in BV2 microglia stimulated by LPS [17]. So we detected the protein levels of TNF-*α*, IL-1*β*, and IL-6 by ELISA. The result shows that the expression of proinflammatory cytokines is induced by hemin stimulation in microglial cells. And the increment is blocked by knockdown of CDK5 (Figures 5(a)–5(c)). It indicates that this function of p-DRP1 depends on CDK5 activity.

The article "CDK5 Mediates Proinflammatory Effects of Microglia through Activated DRP1 Phosphorylation in Rat Model of Intracerebral Hemorrhage" was published in 2022. Journal: Dis Markers.

## 4. Discussion

ICH is a devastating cerebrovascular disease that includes primary injury and secondary injury [1]. Inflammation is an important component of the secondary injury. Recent studies focus on the inflammation after ICH and make an effort to reduce the influence of overactivated microglia [2]. So inhibition of overactivated microglia and secretion of proinflammatory mediators can be an effective therapeutical strategy of ICH.

In recent years, abnormal CDK5 expression is associated with some neurodegenerative or cardiovascular diseases. Specific CDK5 function in microglia was first explored [12]. They found a potential role of the CDK5/p25-LPL signaling pathway in A*β* phagocytosis by microglia and provide a new insight into the molecular pathogenesis of AD [13]. Microglia is the macrophage in central nervous system, and the classic function of microglia is regulating inflammatory reaction [17]. To further explore the connection between CDK5 and microglia, we reveal role of CDK5 in regulating inflammatory reaction in microglia in the ICH model. Mitochondrial fission and fusion are modulated by many genes including dynamin-related protein 1 (Drp1) and mitochondrial fission 1 (Fis1) along with the fusion mediators mitofusin 1 (Mfn1), mitofusin 2 (Mfn2), and optic atrophy 1 (Opa1) [18]. DRP1 especially showed its regulative role in microglia in neuroinflammation [17]. CDK5 and DRP1 have been demonstrated that their interaction can induce mitochondrial fission in neuron [15]. Since CDK5 and DRP1 also play different role in microglia, to probe if their interaction also exist and function in microglia, we detect their interaction and measure proinflammatory mediator secretion with or without knockdown of CDK5 or DRP1. The result shows that CDK5 can phosphorylate DRP1 in microglia, and the phosphorylation of DRP1 promotes microglial cell expression of proinflammatory mediators in the ICH model.

However, our study has its own limitations. Due to the simplicity of the experimental design, some experimental data cannot fully enrich the accuracy of the experimental results. The specific regulatory mechanism between CDK5 and DRP1 has not been deeply explored. Therefore, in the next study, we will further explore the relationship between CDK5 and DRP and the regulatory mechanism, so as to provide an important basis for the pathology of ICH diseases.

The article "CDK5 Mediates Proinflammatory Effects of Microglia through Activated DRP1 Phosphorylation in Rat Model of Intracerebral Hemorrhage" was published in 2022. Journal: Dis Markers.

In a conclusion, our result shows DRP1 as a phosphorylated substrate of CDK5 in microglia, and the phosphorylation of DRP1 promotes the secretion of proinflammatory mediators by microglia in the ICH model. It may provide a therapeutic target of ICH.

## Figures and Tables

**Figure 1:** Neurological deficit score. Forelimb placing (a) and corner turn (b) were scores at different time points following ICH. *N* ≤ 8, ^∗^*p* < 0.05 vs. sham. ICH: intracerebral hemorrhage; d: day.

**Figure 2:** Representative microphotographs for CDK5 immunohistochemistry in the rat brain caudate nucleus around the hematoma: the sham group (brain right caudate nucleus) (a, b); at day 2 after ICH, the contralateral group (contralateral brain tissue of the hematoma) (c, d); the ipsilateral group (brain caudate nucleus adjacent to the hematoma) (e, f). No positive signals in the negative control (g). The number of CDK5 cells in the ipsilateral group compared with the sham and contralateral groups (h). *N* = 5, ^∗^*p* < 0.05 vs. sham. d: day. Scale bar: left columns, 50 *μ*m; right columns, 20 *μ*m.

**Figure 3:** Expression profiles of CDK5 and p35/25 around the hematoma at each time point after ICH by Western blot analysis. Protein expression levels of CDK5 (a). The bar graph indicated the relative density of CDK5 versus *β*-actin at each time point (b). Protein levels of p35/25 (c). Quantification of the increase in p35/25 after ICH (d). *N* = 5, ^∗^*p* < 0.05 vs. sham. ICH: intracerebral hemorrhage; d: day.

**Figure 4:** Expression of p-DRP1 following ICH is dependent on change of CDK5 kinase activity. Protein expression levels of p-histone H1 (a). Quantification of p-histone H1 after ICH (b). The expression of p-DRP1 (c). Quantification of p-DRP1 after ICH (d). Coimmunoprecipitation between CDK5 and DRP1 in microglia, the upper, IP: DRP1, WB: CDK5, and DRP1; the lower, IP: CDK5, WB: DRP1, and CDK5 (e). The expression level of p-DRP1 following knockdown CDK5 or p35 expression by siRNA (f, g). *N* = 5, ^∗^*p* < 0.05 vs. sham. ICH: intracerebral hemorrhage; d: day. IP: immunoprecipitation. “Input” means samples before the IP procedure. “IgG” was used to exclude specific binding. “WB” means Western blot.

**Figure 5:** TNF-*α*, IL-1*β*, and IL-6 expressions in microglial cells in response to stimulus by hemin. The protein levels of TNF-*α*, IL-1*β*, and IL-6 were detected by ELISA (a–c). *N* = 5, ^∗^^,#^*p* < 0.05 vs. sham. h: hour.

The article "CDK5 Mediates Proinflammatory Effects of Microglia through Activated DRP1 Phosphorylation in Rat Model of Intracerebral Hemorrhage" was published in 2022. Journal: Dis Markers.

## Data Availability

The data used to support the findings of this study are available from the corresponding authors upon request.
